RETRACTED

# Thromboelastography Parameters in Urosepsis: A Retrospective Study

**DOI:** 10.1155/2022/9142489

**Published:** 2022-08-17

**Authors:** Yun Qiao, Xiaoye Lu

**Affiliations:** Department of Emergency Medicine, Ren Ji Hospital, Shanghai Jiao Tong University School of Medicine, Shanghai 200127, China

## Abstract

Thromboelastography (TEG) is usually used to monitor coagulation disorder clinically. It is unclear whether TEG has association with urosepsis and sepsis-induced coagulopathy (SIC). The purpose of this study was to investigate the clinical significance of TEG parameters in urosepsis. 90 patients who were admitted to the Emergency Ward and Emergency Intensive Care Unit (EICU) of Ren Ji Hospital affiliated to Shanghai Jiao Tong University School of Medicine due to urinary infection from February 2014 to February 2022 were retrospectively studied. Urosepsis patients and non-sepsis patients were separately investigated according to the final discharge diagnosis and Sepsis 3.0. At the same time, patients with urosepsis were further divided into groups of SIC and non-SIC based on the definition of SIC. The data of clinical features, laboratory biomarkers, and TEG parameters were collected and analyzed. There were significant differences in white blood cell count, C-reactive protein (CRP), platelet count, procalcitonin (PCT), fibrinogen (FIB), international normalized ratio (INR), prothrombin time (PT), D-dimer, and incidence of urinary tract obstruction between the urosepsis group and non-sepsis group (*P* < 0.05). In the comparison with non-sepsis group, K value was significantly lower (*P* = 0.006), while *α*-angle (*P* = 0.003) and clot index (CI) (*P* = 0.048) were significantly higher in urosepsis group. The area under the K value curve excluding urosepsis was 0.667. The areas under CI and *α*-angle curves for diagnosing urosepsis were 0.682 and 0.621, respectively. The patients in SIC group had significantly higher K value, lower *α*-angle, and maximum amplitude (MA) than those in non-SIC group (*P* < 0.05). Coagulopathy is prone to occur in patients with urosepsis. TEG is helpful for assessment of hypercoagulable state in urosepsis and prediction of hypocoagulability in SIC patients implying the dynamic process of DIC.

## 1. Introduction

Emergency department, as the first department to diagnose and treat acute infectious diseases, faces various challenges. Urinary tract infection (UTI) is common in emergency department as a kind of clinically acute infectious disease. If UTI is not diagnosed as early as possible, patients' conditions may deteriorate rapidly, even resulting in sepsis or septic shock. Sepsis is a kind of disease with high incidence and morality. Blood coagulation disorder is common in sepsis. Thromboelastography (TEG) often indicates dynamic coagulation changes and shows underlying clinical value for predicting the dysfunction of blood coagulation for urosepsis patients. Therefore, the study was designed to evaluate the diagnostic value of TEG parameters in urosepsis and sepsis-induced coagulopathy (SIC).

RETRACTED

## 2. Materials and Methods

### 2.1. Subjects

90 patients admitted to Emergency Ward and Emergency Intensive Care Unit (EICU) of Ren Ji Hospital affiliated to Shanghai Jiao Tong University School of Medicine (Shanghai, China) due to urinary tract infection from February 2014 to February 2022 were retrospectively studied. There were 50 females/40 males, with age of 25–94 (72.067 ± 13.679) years. The enrolled patients were divided into two groups: urosepsis and non-sepsis groups, based on the final discharge diagnosis and Sepsis 3.0 [1]. According to the definition of SIC, the urosepsis group was further divided into two subgroups: SIC and non-SIC subgroups [2].

### 2.2. Exclusion Criteria

The patients were excluded if they were under the age of 18, or had underlying conditions as follows: (i) hematological system diseases including congenital coagulant disorders or thromboembolic diseases; (ii) cirrhosis; (iii) terminal state of chronic diseases; (iv) malignant tumor; (v) pregnancy; (vi) pre-existing/receiving medical treatment of antiplatelet or anticoagulant within 2 weeks before admission.

### 2.3. Clinical Data

All blood samples underwent tests in 24 hours after the patients were admitted. Routine blood indexes were determined by the Sysmex XE-2100 automatic blood analyzer. The level of serum procalcitonin (PCT) was detected by double-antibody sandwich immune luminescence with the aid of automatic electrochemical luminescence analyzer (Roche cobas 6000). We used automatic protein analyzer (Siemens BNII) to test the level of serum C-reactive protein (CRP). The indicators of coagulation, such as thrombin time (TT), prothrombin time (PT), activated partial thromboplastin time (APTT), plasma fibrinogen (FIB), D-dimer, and international normalized ratio (INR), were determined with automatic blood coagulation instrument (ACL TOP 700, IL Company). We applied the analyzer for blood coagulation (TEG 5000) to detect TEG indicators, involving *R* time (R), maximum amplitude (MA), K time (K), lysis at 30 min (LY30), time to maximum amplitude (TMA), clot index (CI), *α*-angle, and global clot strength (*G*).

### 2.4. Analysis for Statistics

SPSS 24.0 was applied for data handling. ‾*X*± SD represented statistics of a normal distribution as well as a homogeneity of variance; in addition to that, the remaining data were expressed in the form of median (range), and count data were expressed in the form of frequency (proportion). When comparing differences between groups, the samples with normal distribution of measurement data were analyzed by *t*-test, the samples with non-normal distribution were analyzed by the Mann–Whitney *U* test, and count data were tested by chi-square. TEG parameters were analyzed by ROC curve. In hypothesis testing, if *P* < 0.05, there was a significant difference.

RETRACTED

## 3. Results

### 3.1. Basic Information

45 cases were diagnosed as urosepsis and 45 cases as non-sepsis. SOFA score, white blood cell count, CRP, PCT, and incidence of urinary tract obstruction were significantly increased in the urosepsis group than those in the non-sepsis group (*P* < 0.05), while platelet count was significantly decreased (*P* < 0.05). The comparison results of clinical parameters between two groups are shown in Table 1.

### 3.2. Coagulation and TEG Parameters in Urosepsis and Non-Sepsis Groups

Compared with non-sepsis group, the level of INR, fibrinogen, D-Dimer, CI, and *α*-angle was significantly increased, prothrombin time (PT) was significantly prolonged, and K value was remarkably lower in urosepsis patients (*P* < 0.05). Comparison results of coagulation and TEG parameters between two groups are presented in Table 2.

### 3.3. ROC Curve Analysis for TEG Parameters in Urosepsis Diagnosis

ROC curve analysis was performed for the exclusion of urosepsis at K time, and AUC was 0.667 (95% CI was 0.555 ∼ 0.778). Cutoff value of K time calculated was 1.25 (sensitivity: 64.4%; specificity: 60.0%) (Figure 1). For diagnosing urosepsis, AUC of *α*-angle was 0.682 (95% CI was 0.573 ∼ 0.792), and CI was 0.621 (95% CI was 0.504∼ 0.737). Cutoff value of *α*-angle was 75 (sensitivity: 75.6%; specificity: 57.8%), as shown in Figure 2. Cutoff value of CI calculated was 2.55 (sensitivity: 42.2%; specificity: 84.4%) (Figure 3).

### 3.4. TEG Parameters in Groups of SIC and Non-SIC

13 cases of SIC and 32 cases of non-SIC were enrolled. K time was significantly longer, and *α*-angle and MA value were expressively lower for SIC patients than non-SIC patients (*P* < 0.05).  Table 3 shows the comparison results of TEG parameters between the two groups.

## 4. Discussion

Urosepsis is a kind of sepsis due to the infection of urogenital tract and is regarded as the systemic reaction to infections [3]. Besides, urosepsis often has an acute onset and severe clinical manifestations. If not treated in time, urosepsis can lead to life-threatening conditions. This research showed that urinary tract obstruction diseases were more likely to occur in the urosepsis group. Patients with upper urinary tract infection were prone to develop urosepsis. Obstructive uropathy due to renal stones is a well-known cause of urosepsis [4]. If post-kidney obstruction leads to the ureteral pressure rise, more and more nephrons would stop filtering and produce decreased glomerular filtration with a decline in the urinary concentrations. The process mentioned above can be strengthened based on the obstructed kidney infection, which can lead to urosepsis [5]. If the obstruction is not relieved immediately, acute kidney injury (AKI) caused by post-kidney obstruction can progress to chronic renal failure [6]. Surgical release of urinary tract obstruction is the most effective way to prevent urosepsis even in the absence of sepsis. Our study showed that the concentration of inflammatory markers was increased and the organ dysfunction was more severe in urosepsis patients than non-sepsis patients. There were significant differences in white blood cell count, CRP, PCT, SOFA score, and platelet count between the two groups (*P* < 0.05). Thrombocytopenia caused by urosepsis is also more common and is often detected early. Platelets can rebound after correction of sepsis, and thrombocytopenia may be associated with infection-mediated destruction [7]. Bone marrow suppression may be a factor in some septic patients [8]. Non-catalytic receptors such as toll-like receptors (TLRs) have been suggested as possible mediators of sepsis-associated thrombocytopenia [9]. The endothelial dysfunction caused by sepsis can promote the endogenous coagulation system, resulting in the formation of thrombus and platelet consumption [10]. Therefore, how to quickly and accurately detect whether patients are at risk of hypocoagulable state in clinical practice and timely monitor whether the measures taken are effective is a problem to be solved by our research.

RETRACTED

The disorder of coagulation is frequently seen in sepsis patients. This disease permeates the whole course of sepsis and is a principal element affecting patients' prognosis. TEG can characterize and stimulate the dynamic changes of coagulation and fibrinolysis which plays an increasingly important role in emergency, acutely bleeding trauma, neonatology, and other clinical fields recently [11–13]. Our study showed remarkable difference at K time, *α*-angle, and CI between the two groups. We also found that the urosepsis group had obviously lower K value while *α*-angle and CI of the urosepsis group were increased. K time indicated the speed of blood-clot netting and the *α*-angle reflected clot formation rate, which was mainly influenced by the functions of platelet, thrombin, and fibrinogen. The *α*-angle was closely related to K time and both of them were indicators of the function of fibrinogen, reflecting the rate of clot aggregation [14, 15]. MA value reflected functions of platelet aggregation and CI reflected the comprehensive coagulation state of blood sample. Significant difference was not found between the two groups in MA value. CI was an index calculated from all TEG parameters and was better than MA value [14], which indicated that patients with urosepsis were in a hypercoagulable state compared with those without sepsis. The specificity of CI in our study was more than 80%, indicating CI had better diagnostic value for early stage of urosepsis [16]. These TEG parameters were correlated with each other and can be widely used to predict the coagulation state of patients from all aspects in clinic [17–19]. During sepsis, under the action of bacteria and endotoxins, vascular endothelial cells (VEC) were stimulated, platelet aggregation was activated, and coagulation factors, cytokines, and vasoactive substances were released, which facilitated the formation of microthrombosis and the inhibition of anticoagulation system and fibrinolytic system [20]. Zhou et al. found that indicators, including CI, *α*-angle, MA value, *R* value, and K time, can facilitate determination of condition severity in patients [14]. Anticoagulant therapy can predict the likely future course and outcomes of the disease and has the potential to lower the death rate in patients with sepsis [21]. Appropriate target selection and early, rapid diagnosis of sepsis are essential for anticoagulant treatment [22].

The values of PT, INR, FIB, and D-dimer showed differences in patients with urosepsis and non-sepsis (*P* < 0.05). Hyperfibrinogenemia in the process of sepsis was the result of hepatic protein metabolism toward the predominant synthesis of pro-inflammatory proteins [23], and elevated D-dimer indicated the hypercoagulable state of patients with urosepsis. A recent study indicated that INR was most effective in diagnosing non-pulmonary infectious sepsis, when an INR value above 1.22 was achieved in patients with infections not located in the lungs [16]. A new scoring system, including INR, platelet count, and SOFA score, was proposed to define sepsis-induced coagulopathy (SIC) [2]. Disseminated intravascular coagulation (DIC) refers to systemic activation of intravascular coagulation due to various causes [24]. SIC continues from an initial compensatory phase to the decompensated phase of DIC in patients with sepsis, including the hemorrhagic and thrombotic state [25]. Koami et al. reported that TEG was a single reliable indicator of sepsis-induced DIC and was strongly associated with severity of DIC [26]. Besides, we assessed their diagnostic value of TEG parameters with respect to SIC as well as the relation of TEG to SIC. SIC group showed obviously higher K value than the group of non-SIC, and at the same time, *α*-angle and MA value in SIC group presented lower values than non-SIC group (*P* < 0.05). Prolonged K time and reduced *α*-angle and MA value indicated that patients in the SIC group were in a hypocoagulable state. Luo et al. found that K time had high accuracy in diagnosing SIC, and *α*-angle and MA values had high accuracy in excluding SIC [27]. A recent study showed that in terms of *R* time and *α*-angle, the mortality of patients in hypocoagulable states was higher than that of patients with normal coagulation [28], indicating that hypocoagulable state was closely related to patients' prognosis. The size of samples in the study was comparatively small, and therefore, the statistical power was limited. The relation of SIC to TEG needs to be further studied.

RETRACTED

In summary, thromboelastography may have diagnostic value for urosepsis and indicate distinct changes of coagulation in patients with urosepsis. TEG measurements may be better than routine tests in judging the blood coagulation disorder of urosepsis. Furthermore, TEG may reflect the hypocoagulable state of patients and help predict sepsis-induced coagulopathy.

## Figures and Tables

**Figure 1:** ROC curve analysis of K time for urosepsis diagnosis.

**Figure 2:** ROC curve analysis of *α*-angle for urosepsis diagnosis.

**Figure 3:** ROC curve analysis of CI for urosepsis diagnosis.

**Table 1:** Clinical parameters in patients between two groups.

Items	Urosepsis group	Non-sepsis group	*P*
	*n* = 45	*n* = 45	
Gender (male, %)	19 (42.22)	21 (46.67)	0.671
Age (years)	74.600 ± 13.491	69.533 ± 13.541	0.079
SOFA	3 (2, 5)	0 (0, 1)	0.000^*∗*^
White blood cell (×10^12^)	11.160 (6.940, 17.835)	7.120 (5.615, 10.930)	0.003^*∗*^
Platelets (×10^9^)	138.000 (92.500, 188.000)	181.000 (159.500, 265.500)	0.000^*∗*^
C-Reactive protein (mg/L)	117.880 (73.910, 182.230)	38.850 (17.400, 109.740)	0.000^*∗*^
Procalcitonin (*μ*g/L)	3.700 (0.735, 32.295)	0.250 (0.100, 1.355)	0.000^*∗*^
Urinary irritation (%)	9 (20.00)	13 (28.89)	0.327
Urinary tract obstruction (%)	16 (35.56)	7 (15.56)	0.030^*∗*^
Indwelling catheter (%)	5 (11.11)	5 (11.11)	1.000
Acute pyelonephritis (%)	7 (15.56)	5 (11.11)	0.535
History of urologic surgery	5 (11.11)	5 (11.11)	1.000

**Table 2:** Comparative results of routine coagulation indicators and TEG parameters in patients between two groups.

Items	Group of urosepsis	Group of non-sepsis	*P*
	*n* = 45	*n* = 45	
PT (s)	13.000 (11.850, 14.150)	11.900 (10.750, 12.750)	0.000^*∗*^
APTT (s)	30.900 (28.000, 33.050)	29.700 (27.400, 32.250)	0.194
TT (s)	16.300 (15.100, 17.650)	16.200 (14.600, 17.850)	0.974
FIB (g/l)	4.980 (4.395, 6.590)	4.260 (3.620, 5.860)	0.005^*∗*^
INR	1.140 (1.050, 1.255)	1.080 (0.970, 1.135)	0.000^*∗*^
D-Dimer (*μ*g/ml)	1.060 (0.805, 2.310)	0.520 (0.300, 1.135)	0.000^*∗*^
R (min)	6.200 (5.350, 7.150)	6.700 (5.850, 7.300)	0.093
K (min)	1.200 (1.000, 1.500)	1.500 (1.200, 1.800)	0.006^*∗*^
*α*-Angle (deg)	75.200 (70.650, 78.300)	71.500 (67.200, 75.350)	0.003^*∗*^
MA (mm)	67.942 ± 7.488	67.242 ± 5.780	0.621
CI	1.900 (0.700, 3.050)	1.200 (-0.100, 2.300)	0.048^*∗*^
LY30 (%)	0 (0, 0)	0 (0, 0)	0.498
G (d/sc)	11464.596 ± 4075.792	10711.576 ± 2677.610	0.303
TMA (min)	25.522 ± 3.760	27.091 ± 4.120	0.063

RETRACTED

**Table 3:** Comparison results of TEG parameters between the group of SIC and the group of non-SIC.

Items	SIC group	Non-SIC group	*P*
	*n* = 13	*n* = 32	
SIC score	5 (4, 5)	2 (2, 3)	0.000^*∗*^
R (min)	6.100 (5.150, 7.800)	6.200 (5.325, 7.075)	0.783
K (min)	1.600 (1.050, 2.000)	1.200 (1.000, 1.400)	0.045^*∗*^
*α*-Angle (deg)	70.600 (66.300,76.300)	76.000 (73.050, 78.750)	0.023^*∗*^
MA (mm)	64.315 ± 7.831	69.416 ± 6.935	0.037^*∗*^
CI	1.000 (−0.850, 2.850)	2.150 (0.925, 3.175)	0.101
LY30 (%)	0 (0, 0)	0 (0, 0)	0.259
G (d/sc)	9670.092 ± 3405.555	12193.613 ± 4146.074	0.059
TMA (min)	27.039 ± 4.350	24.906 ± 3.375	0.085

## Data Availability

The simulation experiment data used to support the findings of this study are available from the corresponding author upon request.
